# Application Effect of Cluster-Based Care in Patients with Hypertensive Disorders of Pregnancy and Osteoarthritis

**DOI:** 10.1155/2022/2954330

**Published:** 2022-08-04

**Authors:** Lili Ye, Chunhua Yu, Xiaoqin Chen, Yanyan Han

**Affiliations:** ^1^Department of Spine Surgery, Chengyang District People's Hospital of Qingdao City, Qingdao 266109, China; ^2^Department of Gynecology, Chengyang District People's Hospital of Qingdao City, Qingdao 266109, China; ^3^Department of Obstetrics, Chengyang District People's Hospital of Qingdao City, Qingdao 266109, China

## Abstract

**Objective:**

To explore the application effect of cluster-based care in patients with hypertensive disorders of pregnancy and osteoarthritis.

**Methods:**

The clinical data of 60 patients with hypertensive disorders of pregnancy and osteoarthritis in our hospital were retrospectively analyzed, among which those receiving routine care from January 2020 to December 2020 were grouped into the control group (30 patients), and those receiving cluster-based care from January 2021 to January 2022 were grouped into the research group (30 patients). Psychological status, care satisfaction, and pregnancy outcomes were compared between the two groups.

**Results:**

After intervention, self-rating anxiety scale (SAS) and self-rating depression scale (SDS) scores in the research group were lower than those in the control group (*P* < 0.05). There was no statistical significance in the difference of the modes of delivery between the two groups (*χ*^2^ = 1.763, *P* > 0.05). Patients in the research group had a lower incidence of perinatal complications than those in the control group (*χ*^2^ = 5.689, *P* < 0.05). And the satisfaction rate of care in the research group (93.33% vs 70%) was higher than that in the control group (*χ*^2^ = 4.238, *P* < 0.05).

**Conclusion:**

Cluster-based care can reduce patients' negative mood, increase their satisfaction, and improve the maternal and infant outcomes. This type of care offers better quality care measures for patients with pregnancy hypertension and osteoarthritis, and has a wide clinical application prospect.

## 1. Introduction

Hypertensive disorder of pregnancy is a common condition during pregnancy. It includes eclampsia and preeclampsia and is a common disease in obstetrics and gynecology clinics [1]. Parturients with hypertensive disorders of pregnancy have a much greater risk of postpartum hemorrhage than normal parturients, and complicated osteoarthritis will further reduce parturients' limb mobility and affect their maternal physical and mental health [2, 3]. Therefore, in clinical practice, nursing staff must improve the attention on hypertensive disorders of pregnancy with osteoarthritis. Cluster-based care is a kind of advanced care concept based on Nightingale's modern care positioning as “the patient-centered delivery of high-quality care.” Cluster emphasizes to improve the degree of humanistic care for patients, patients' satisfaction, and prognosis quality through a series of physiological and psychological evidence-based care measures [4, 5]. This study adopted cluster-based care as the intervention for patients with hypertensive disorders of pregnancy and osteoarthritis, to explore the effect of cluster-based care on patients' negative emotions and compare satisfaction and infant pregnancy outcomes across different care models, which is reported as follows.

## 2. Data and Methods

### 2.1. General Data

The clinical data of 60 patients with hypertensive disorders of pregnancy and osteoarthritis receiving the treatment in our hospital from January 2020 to January 2022 were retrospectively analyzed, among which those receiving routine care from January 2020 to December 2020 were grouped into the control group (30 patients), and those receiving cluster-based care from January 2021 to January 2022 were grouped into the research group (30 patients). Inclusion criteria are as follows: ① patients who met the diagnostic criteria for hypertensive disorders of pregnancy [6]; ② patients who met the diagnostic criteria for osteoarthritis [7]; ③ patients who underwent labor examination and delivery in our hospital; and ④ patients with singleton pregnancy, who had been informed and voluntarily participated in the study. Exclusion criteria are as follows: ① patients with maternal age < 20 years; ② patients with other gestational syndromes (such as gestational hypothyroidism, and gestational diabetes); and ③ patients with immunodeficiency disease. This study has been approved by the ethics committee of Chengyang District People's Hospital, and informed consent was obtained from all patients.

### 2.2. Methods

Parturients in the control group were given the maternal routine care intervention, who were then guided for prenatal examination with their families, and were carried out health education and psychological counseling during perinatal period, to reduce their stress response and psychological negative emotions. Before and after delivery, the basic vital signs of parturients were routinely monitored, the risk of postpartum hemorrhage was assessed, and parturients were given uterine floor massage to promote contractions. Research group accepted cluster-based care. ① Psychological care: Specialized nurses monitored the psychological state of parturients every day and assessed their negative emotions through communication with them and their behaviors or movements. Direct accompaniment, health education, chat to divert attention, and other ways were adopted to reduce the psychological burden of parturients; at the same time, the family member were urged to actively accompany and give full social and family support to the parturients. ② Dietary care and blood pressure monitoring: Specialized nurses provided dietary guidance and blood pressure monitoring to the parturients every day, among which the blood pressure was monitored 4 times a day, and the diet was mainly liquid food that is easy to digest, high in fiber and light. When the blood pressure was higher than the ideal value, the doctor was informed immediately and symptomatic intervention was given. ③ Position care: During the perinatal period, the maternal position management was strengthened to reduce the chance of maternal bleeding. Before cesarean section, the parturients were fully rested in bed to avoid getting out of bed at will. Meanwhile, the left lying position was used to reduce the risk of maternal bleeding and the impact on the fetus. ④ Limb function exercise: Hypertensive disorders of pregnancy complicated with osteoarthritis can seriously reduce the maternal capacity for limb movement and increase the risk of microcirculation disorders. Therefore, nurses guided parturients for appropriate intensity of physical activity to promote the recovery of limb functions and prevent the formation of local thrombosis. The training movements were mainly light exercises such as finger, wrist, elbow, knee, and toe joint exercises to avoid increasing the physical and mental burden of parturients. ⑤ Prevention of postpartum hemorrhage: Before and after delivery, the situation of vaginal bleeding of parturients was continuously monitored, and at the same time, ECG monitoring was carried out to observe the contraction of uterus after child's birth, the height of fundus uteri, the intestinal bladder filling, the perineum, and the vagina that have hematomas. In case of any abnormal condition, special gauze was used in time for uterine tamponade to initially stop bleeding and immediately inform the attending physician.

### 2.3. Observational Indexes

(1) Psychological status: SAS [8] and SDS [9] scores were compared between the two groups before and after intervention. Both scales had 20 items, with the total score of 80 points. The higher the score was, the more serious the anxiety or depression was. (2) Maternal and infant outcome indexes: The mode of delivery and the occurrence of preterm labor, puerperal infection, and postpartum hemorrhage were compared between the two groups. (3) Care satisfaction: Before maternal discharge, self-made satisfaction questionnaires in our department were used to collect patients' and family members' satisfaction data, and based on the score of the questionnaire, it was divided into very satisfied (≥85 points), basically satisfied (70~84 points), unsatisfied (<70 points), and overall satisfied = very satisfied + basically satisfied.

### 2.4. Statistical Method

Data were analyzed by SPSS 22.0.The measurement data were represented by ($\bar{\text{x}}\pm \text{s}$), and *t*-test was used for comparison between the two groups. The count data is expressed by *n* (%) and verified by *χ*^2^ test. A *P* value < 0.05 was considered statistically significant.

## 3. Results

### 3.1. Comparison of Baseline Data between the Two Groups

The differences in age (*t* = 0.626), gestational age (*t* = 0.298), body mass index (*t* = 0.241), and history of pregnancy (*χ*^2^ = 0.268) of the two groups were have no statistical significance (*P* > 0.05), as shown in Table 1.

### 3.2. Comparison of Psychological Status between the Two Groups

There was no statistically significant difference in SAS and SDS scores before the intervention compared to the two groups (*P* > 0.05). SAS (*t* = 10.792) and SDS (*t* = 11.570) scores in the research group were lower than those of the control group after intervention (*P* < 0.05), as shown in Table 2.

SAS: self-rating anxiety scale; SDS: self-rating depression scale.

### 3.3. Comparison of Maternal and Infant Outcomes between the Two Groups

There was no significant difference in the mode of delivery between the two groups (*χ*^2^ = 1.763, *P* > 0.05). The rate of perinatal complications was lower in the research group than in the control group (*χ*^2^ = 5.689, *P* < 0.05), as shown in Table 3.

### 3.4. Comparison of Satisfaction between the Two Groups

The satisfaction of care in the research group (93.33% vs 70%) was higher than that of the control group (*χ*^2^ = 4.238, *P* < 0.05), as shown in Table 4.

## 4. Discussion

The incidence of serious complications in pregnant women and parturients with hypertensive disorders of pregnancy is high and harmful, which will increase the risk of postpartum hemorrhage, affect the outcomes of pregnancy, and even endanger the life safety of mother and baby in serious patients. The pathogenesis of hypertensive disorders of pregnancy is complicated. Clinical studies [10–12] pointed out that the occurrence of this disease may be related to placenta, maternal underlying disease, or mood abnormalities. Abnormal elevated blood pressure is the main clinical feature of hypertensive disorders of pregnancy. If prenatal treatment intervention cannot be given in time, it may lead to abortion. Hypertensive disorders of pregnancy is an independent risk factor for postpartum bleeding, and osteoarthritis will lead to further reduction of patients' daily activities, affecting the daily life of patients [13, 14]. The traditional mode of care can mainly reduce the risk of pregnancy through prenatal examination guidance, blood pressure control, health education, and medication guidance. However, due to the lack of refined and targeted nursing measures in traditional care, the actual nursing needs of patients are ignored, so it is difficult to achieve satisfactory care effect.

The results of this study showed that SAS score and the rate of perinatal complications in the research group were lower than that in the control group, indicating that cluster-based care can improve the negative mood and reduce the risk of complications in patients with hypertensive disorders of pregnancy and osteoarthritis, which are similar to the study of Xiao et al. [15]. The results also showed that the nursing satisfaction (93.33% vs 70%) in the research group was higher than that in the control group, which is corresponding to the study of Di et al. [16], indicating that cluster-based care can improve the care satisfaction of patients with hypertensive disorders of pregnancy and osteoarthritis. According to the analysis on the reasons, this is due to the targeted evidence-based psychological intervention measures to improve the maternal psychological negative mood, including dietary care, blood pressure monitoring, body care, physical function exercise, and postpartum bleeding prevention; reduce the risk of perinatal complications; and improve patient satisfaction. Our study also has some limitations. Insufficient sample size was included in the study, and the reliability of the results was not strong, and we further expand the sample size to verify our conclusions. The clinical observation indexes in the study were too few, and we should increase the observation indexes in future studies.

In conclusion, cluster-based care has good results in patients with hypertensive disorders of pregnancy and osteoarthritis, which can reduce patients' negative emotions, increase patient satisfaction, improve maternal and infant pregnancy outcomes, and has clinical promotion value.

## Figures and Tables

**Table 1:** Comparison of baseline data between the two groups.

Group	*n*	Age (years old)	Pregnancy age (weeks)	Body mass index (kg/m^2^)	Pregnancy history (*n* (%))	
					Primiparity	Multiparity
Research group	30	30.35 ± 4.15	36.41 ± 5.12	22.35 ± 4.15	17 (56.67)	13 (33.33)
Control group	30	29.89 ± 3.89	36.68 ± 4.80	22.17 ± 4.02	15 (50.00)	15 (50.00)
*t*/*χ*^2^		0.626	0.298	0.241	0.268	
*P*		0.532	0.766	0.810	0.605	

**Table 2:** Comparison of psychological status of the two groups ($\bar{\text{x}}\pm \text{s}$, points).

Group	*n*	SAS		SDS	
		Before intervention	After intervention	Before intervention	After intervention
Research group	30	52.35 ± 4.26	15.33 ± 3.59	45.14 ± 5.30	18.59 ± 2.61
Control group	30	51.47 ± 4.11	25.52 ± 4.28	44.83 ± 5.13	27.27 ± 3.59
*t*		0.880	10.792	0.249	11.570
*P*		0.382	<0.001	0.804	<0.001

**Table 3:** Comparison of maternal and infant outcomes between the two groups (*n* (%)).

Group	*n*	Mode of delivery		Perinatal complications			
		Natural labor	C-sect	Premature birth	Puerperal infection	Postpartum hemorrhage	Total complications
Research group	30	16 (53.33)	14 (46.67)	2 (6.67)	0	1 (3.33)	3 (10.00)
Control group	30	21 (70.00)	9 (30.00)	6 (20.00)	2 (6.67)	4 (13.33)	12 (40.00)
*χ* ^2^		1.763					7.200
*P*		0.184					0.007

**Table 4:** Comparison of satisfaction between the two groups (*n* (%)).

Group	*n*	Very satisfied	Basically satisfied	Unsatisfied	Satisfaction of care
Research group	30	20 (66.67)	8 (26.67)	2 (6.67)	28 (93.33)
Control group	30	11 (36.67)	10 (33.33)	9 (30.00)	21 (70.00)
*χ* ^2^					5.455
*P*					0.020

## Data Availability

The simulation experiment data used to support the findings of this study are available from the corresponding author upon request.
